# Curative Effect of Yangxin Dingji Capsule Combined With Mexiletine Hydrochloride on Postoperative Arrhythmia and Its Influences on the Vascular Endothelial Function in Coronary Bifurcation Lesions

**DOI:** 10.1155/2022/4078895

**Published:** 2022-08-30

**Authors:** Nasha Sun, Wangkun Chen, Yan Wu, Qiyi Yu, Xia Zhou, Bing Guo

**Affiliations:** ^1^Department of Clinical Pharmacy, Ningbo Yinzhou No. 2 Hospital, Ningbo, Zhejiang 315100, China; ^2^Department of Encephalopathy, Wuxi No. 2 Chinese Medicine Hospital, Wuxi, Jiangsu 214121, China; ^3^Department of Science and Education Section, Wuxi No. 2 Chinese Medicine Hospital, Wuxi, Jiangsu 214121, China; ^4^Department of Cardiovascular Medicine, Wuhan Caidian District People's Hospital, Wuhan, Hubei 430100, China

## Abstract

**Objective:**

The aim of the study is to explore the curative effect of Yangxin Dingji capsule combined with mexiletine hydrochloride on postoperative ventricular arrhythmia (VA) and its influences on vascular endothelial function in coronary bifurcation lesions (CBL).

**Methods:**

A total of 110 patients with CBL admitted to the hospital were enrolled as research subjects between January and December 2021. According to the random number table method, they were divided into a combination group and control group, with 55 cases in each group. The control group was treated with mexiletine hydrochloride, while the combination group was additionally treated with Yangxin Dingji capsules. All were continuously treated for 4 weeks. The clinical response rate between the two groups was compared. The frequencies of 24 h paroxysmal atrial fibrillation, premature atrial contraction, and premature ventricular contraction were compared by the Holter monitoring. The whole blood low-shear viscosity, whole blood high-shear viscosity, and fibrinogen (Fb) in both groups were measured by a full-automatic blood flow analyzer. The levels of plasma nitric oxide (NO), endothelin-1 (ET-1), and von Willebrand factor (vWF) were detected by the nitrate reductase method and enzyme-linked immunosorbent assay (ELISA). During treatment, the occurrence of adverse reactions (vomiting, loss of appetite, dry mouth, diarrhea, nausea) in both groups was statistically analyzed.

**Results:**

After treatment, the total response rate of treatment in the combination group was significantly higher than that in the control group (*P* < 0.05). After treatment, frequencies of paroxysmal atrial fibrillation, premature atrial contraction, and premature ventricular contraction in the combination group were significantly lower than those in the control group (*P* < 0.05). Whole blood low-shear viscosity, whole blood high-shear viscosity, and the Fb level were significantly lower than those in the control group (*P* < 0.05). After treatment, the NO level in the combination group was significantly higher than that in the control group (*P* < 0.05), while levels of ET-1 and vWF were significantly lower than those in the control group (*P* < 0.05). During treatment, there was no significant difference in the total incidence of adverse reactions between the two groups (*P* > 0.05).

**Conclusion:**

Yangxin Dingji capsule combined with mexiletine hydrochloride can significantly improve clinical effects in CBL patients, improve VA and vascular endothelial function, and reduce plasma viscosity without increasing the incidence of adverse reactions.

## 1. Introduction

Coronary bifurcation lesions (CBL) are considered to be a coronary stenosis disease and percutaneous coronary intervention (PCI) is often used in clinical practice, and ventricular arrhythmia (VA) often occurs after surgery [1]. Mexiletine hydrochloride is a class Ib sodium channel blocker. It can reduce the depolarization speed of action potential by inhibiting the influx of Na+ in cardiomyocytes to achieve the purpose of treating VA, but long-term use will cause vomiting and nausea in patients. Symptoms such as the abnormal liver function and ventricular rapid heart rate aggravate the patient's VA condition and affect the prognosis [2]. Yangxin Dingpai Capsule belongs to a kind of Chinese patent medicine. It has the functions of calming palpitations, restoring pulse, invigorating qi, nourishing blood, etc. It can exert an anti-VA effect by reducing premature ventricular contraction and has been used for various factors causing VA. The effect is remarkable [3]. Previous studies have found that Yangxin Dingji Capsules combined with Western medicine are significantly more effective than pure Western medicine in the treatment of VA and improve the vascular endothelial function and can also reduce the risk of abnormal heart rate caused by long-term use of Western medicine [4]. At present, the application of mexiletine hydrochloride combined with Yangxin Dingji Capsules in postoperative CBL patients is still in its infancy, and relevant reports are rare. In this study, patients with postoperative CBL were treated with mexiletine hydrochloride combined with Yangxin Dingji Capsules, and the effects on VA and vascular endothelial function were observed. The purpose of this study is to provide some ideas and suggestions for the selection of effective clinical treatment plans in the future.

## 2. Materials and Methods

### 2.1. General Information

A total of 110 CBL patients admitted to our hospital from January 2021 to December 2021 were selected as the research subjects, and they were randomly divided into the combined group and the control group, with 55 cases in each group. Inclusion criteria are as follows: (1) all patients met the CBL-related diagnostic criteria in “Interventional Treatment of Coronary Artery Bifurcation Lesions” [5]; (2) there were no detours or severe calcification in branch or main blood vessels; (3) all patients were included in the study, in line with PCI indications; (4) all patients had arrhythmias after ECG detection; (5) this study was approved by the patients and their families, and was approved by the Medical Ethics Committee of our hospital. Exclusion criteria are as follows: (1) combined with other malignant tumors; (2) suffering from autoimmune diseases; (3) allergic to mexiletine hydrochloride or Yangxin Dingji capsule; and (4) patients with serious abnormal mental and cognitive functions. Control group: 25 males and 30 females; aged 40–71 years, mean (58.88 ± 5.21) years old; body mass index (BMI) 21–28 kg/m^2^, mean (24.67 ± 2.03) kg/m^2^. Medina classification: 27 cases of type 1, 1, 1, and 11 cases of type 0, 1, and 1, and 17 cases of type 1, 0, and 1. Combined group: 28 males and 27 females; age 41–70 years old, mean (57.78 ± 5.55) years old; BMI 22–28 kg/m^2^, mean (24.51 ± 2.33) kg/m^2^. Medina classification: 1 and 1. There were 25 cases of type 1, and 12 cases of type 0, 1, and 1, and 18 cases of type 1, 0, and 1. There was no significant difference in general data such as gender, age, BMI, and Medina classification between the two groups (*P* > 0.05), and the results were comparable.

### 2.2. Methods

Both groups of patients were given basic treatments such as improving coronary circulation and anticoagulation after the operation. At the same time, the control group was given mexiletine hydrochloride (Shanghai Shanghai Pharmaceutical Xinyi Pharmaceutical Co., Ltd., H31021874, 50 mg/tablet). Patients take oral administration in the morning, middle, and evening, 3 times/d, 150 mg/time. The initial dose is 300–500 mg/d. The maximum daily dose cannot exceed 800 mg.

On the basis of the control group, the combined group was given Yangxin Dingji Capsule (Hebei Yongfeng Pharmaceutical Co., Ltd., Z19991082, 500 mg/capsule). Patients take orally in the morning and evening, 2 times/d, 6 capsules/time. Both groups were treated for 4 consecutive weeks.

### 2.3. Observation Indicators

(1) After 4 weeks of treatment, the clinical efficacy evaluation was carried out with reference to the relevant basis in the Guidelines for Clinical Research of New Chinese Medicines [5]. The main clinical symptoms of the evaluation were chest tightness and fatigue, palpitations, shortness of breath, dizziness, and insomnia, and the number of arrhythmias was recorded by an electrocardiogram. All clinical symptoms of the patient were significantly improved, and the number of arrhythmias was reduced by more than 90%.The number of arrhythmias reduced by less than 50% is invalid. The total clinical effective rate = (markedly effective + effective)/total number of patients × 100%. (2) Before the treatment and after 4 weeks of treatment, the patients were observed with a dynamic ECG monitor (HWM-112W, Xuzhou Capital Medical Equipment Co., Ltd.) for 24 hours, and the occurrence of paroxysmal atrial fibrillation and atrial fibrillation in the patients within 24 hours was recorded. The number of premature contractions and ventricular premature contractions occurred, and the VA status of the patients was compared. (3) Before treatment and after 4 weeks of treatment, an automatic blood flow analyzer (XT-1800i, Sysmex Medical Electronics Co., Ltd.) was used to analyze the whole blood low-shear viscosity value, whole blood high-shear viscosity value, fibrinogen (Fb) levels were measured. (4) Before treatment and after 4 weeks of treatment, the serum levels of nitric oxide (NO) and endothelin-1 in the two groups of patients were measured by a nitrate reductase method and enzyme-linked immunosorbent assay (ELISA). (endothelin 1, ET-1) and von Willebrand factor (vWF) levels were detected. Both groups of patients underwent fasting venous blood draw of 4–5 mL in the early morning, and the serum was separated by centrifugation (3000 rpm, 8 cm, 10 min). The samples to be tested were stored in a −20°C refrigerator, and then, the NO detection kit (Guangzhou Jiashengkang Biotechnology Co., Ltd.) and ELISA were used. The levels of NO, ET-1, and vWF were measured by the kit (Shanghai Enzyme Research Biotechnology Co., Ltd.), and the operations were carried out in strict accordance with the kit instructions. (5) During the treatment period, the total incidences of adverse reactions such as vomiting, loss of appetite, dry mouth, diarrhea, and nausea were counted in the two groups.

### 2.4. Statistical Methods

SPSS 22.0 software was used for statistical analysis of the data. The measurement data were expressed as ($\bar{x}$ ± *s*), and the differences in measurement data between groups were compared using an independent *t* test. Differences in measurement data within groups were compared using a paired *t* test. The count data are expressed in (n (%)). A chi-square comparison test was used. Statistical significance was indicated by *P* < 0.05.

## 3. Results

### 3.1. Comparison of Clinical Effects between the Two Groups of Patients

After 4 weeks of treatment, the total clinical effective rate in the combination group was 87.27%, which was significantly higher than that in the control group (69.09%) (*χ*^2^ = 5.329, *P*=0.021) as shown in Table 1.

### 3.2. Comparison of Arrhythmia between the Two Groups

Before treatment, there were no significant differences in the number of paroxysmal atrial fibrillations, atrial pre-systole, and ventricular pre-systole between the two groups (*P* > 0.05). The number of contractions and premature ventricular contractions were significantly lower than those before treatment, and the combined group was significantly lower than the control group (*P* < 0.05) as shown in Table 2.

### 3.3. Comparison of Plasma Viscosity between the Two Groups

Before treatment, there was no significant difference in whole blood low-shear viscosity value, whole blood high-shear viscosity value, or Fb level between the two groups (*P* > 0.05). The viscosity value and Fb level were significantly lower than those before treatment, and the combined group was significantly lower than the control group (*P* < 0.05) as shown in Table 3.

### 3.4. Comparison of Serum NO, ET-1, and vWF Levels between the Two Groups of Patients

Before treatment, there was no significant difference in the levels of NO, ET-1 and vWF between the two groups (*P* > 0.05); after 4 weeks of treatment, the levels of NO in the two groups were significantly higher than those before treatment, and the levels of ET-1 and vWF were significantly lower than those after treatment before, and the level of the combined group was significantly better than that of the control group (*P* < 0.05) as shown in Table 4.

### 3.5. Comparison of Adverse Reactions between the Two Groups of Patients

During the treatment, the total incidence of adverse reactions such as vomiting, loss of appetite, dry mouth, diarrhea, and nausea in the combined group was significantly lower than that in the control group (*P* < 0.05) as shown in Table 5. All patients received corresponding nursing care and treatment when adverse reactions occurred and the symptoms were gradually relieved and disappeared.

## 4. Discussions

PCI is a common surgical procedure for the treatment of CBL in clinical practice. It uses a catheter to dredge occluded or extremely narrowed coronary arteries. It has the advantages of a good curative effect and little damage. At present, western medicines such as mexiletine hydrochloride are often used in the clinical treatment of VA. Although there is a certain curative effect, in the long run, it will have side effects on the function of the kidneys and liver of the patients, which will lead to the rapid ventricular heart rate of the patients. Studies have found that the combined use of traditional Chinese and Western medicines can largely improve VA and vascular endothelial function in patients with high safety [7].

The results of this study showed that the clinical efficacy of the combined group was significantly better than that of the control group, indicating that the use of Yangxin Dingji Capsules combined with western medicine could further improve the clinical efficacy of CBL patients. Traditional Chinese medicine believes that VA is mainly caused by the obstruction of blood vessels, which can be treated by removing the blood vessels. Yangxin Dingpai Capsule is a kind of Chinese patent medicine often used in clinical practice. The specific medicinal ingredients are red ginseng, cinnamon, ginger, roasted licorice, *Rehmannia glutinosa*, *Ophiopogon japonicus*, etc. The roasted licorice is a royal medicine, which has the effects of dredging blood vessels, nourishing blood, and nourishing yin. Among them, red ginseng, *Rehmannia glutinosa*, and *Ophiopogon japonicus* are used as ministerial medicines, which have the functions of nourishing blood and invigoration. With cinnamon twig and ginger as adjuvants, it has the functions of warming the blood and dispersing the acrid; the combination of multiple drugs can play a role in nourishing the blood, nourishing yin, and reconciling yin and yang [8]. Mexiletine hydrochloride can improve VA by regulating the functions of various myocardial ion channels, and the combined use of the two may have a synergistic effect of improving VA. Abnormal activation of the sinus node is the main factor in the production of VA. Paroxysmal atrial fibrillation, premature atrial contractions, and an abnormally increased number of premature ventricular contractions are common clinical features of VA, which can reflect the severity of VA to a certain extent [9]. Therefore, we conducted statistics on the above three indicators in the two groups of patients, and the results found that the reduction of each index in the combination group was greater than that in the control group after treatment, indicating that compared with mexiletine hydrochloride alone, the combined use of Yangxinding Ji Capsules can better improve postoperative arrhythmia in CBL patients to a certain extent. The results of this study are similar to those of Yaning et al. [10] Analysis of the reason may lie in the Zhigancao and Guizhi contained in the Yangxin Dingpal Capsule. Zhigancao contains glycyrrhetinic acid. Glycyrrhetinic acid can promote the increase of ATPase activity in myocardial tissue and ensure that K+ and Na+ in myocardial cells are normal. To inhibit the concentration of Ca2+, thereby reducing the automaticity of cardiac ectopic pacemakers, to achieve the purpose of improving VA. The two most effective components in cinnamon twig are cinnamic acid and cinnamic aldehyde, both of which can prolong the action potential very well, thereby inhibiting cell autonomicity, and finally reducing the abnormal excitation of the sinoatrial node to improve VA.

The increase in whole blood low-shear viscosity value, whole blood high-shear viscosity value, and Fb level indicates that the blood viscosity is increasing, and the microcirculation of the body's blood will also be hindered, resulting in insufficient blood supply and eventually leading to VA [11]. The results of this study showed that the plasma viscosity of the combined group was significantly lower than that of the control group after treatment. The results of this study are partially similar to those of Yaning et al. [12]. The reason may be that the raw *Rehmannia*, licorice, red ginseng and other medicinal ingredients in the Yangxin Dingpal Capsule can promote blood circulation and significantly improve myocardial hypoxia tolerance, thus improving the abnormal state of blood rheology and reducing viscosity. In blood vessels, NO and ET-1 are a pair of main active substances. The rise of ET-1 can cause severe vasoconstriction, while the synthesis of NO by vascular endothelial cells (VEC) has an inhibitory function on ET-1. The dynamic balance between vascular and vascular tone plays an important role in maintaining vascular tone. The increase of vWF can cause thrombosis, and its level will increase significantly when the vascular endothelial function is damaged [13]. The results of this study showed that the improvement of NO, ET-1, and vWF in the combined group was significantly better than that in the control group after treatment. The results of this study by Yaning et al. [14] and others found similar results in patients with acute coronary syndrome (ACS). It shows that Yangxin Dingji Capsules can help improve the vascular endothelial function of CBL patients after surgery. The reason may be that the ginger in Yangxin Dingji Capsules promotes the production of NO from VEC through its effective parts, thereby reducing vascular endothelial damage. *Ophiopogon japonicus* and *Ophiopogon saponin* D inhibit VEC apoptosis and damage by regulating VEC-related functional genes, and the combined action of the two has a good protective effect on vascular endothelial function. There was no significant difference in adverse reactions between the two groups of patients during treatment.

In conclusion, Yangxin Dingji Capsules combined with mexiletine hydrochloride can effectively improve postoperative clinical efficacy, arrhythmia, and vascular endothelial function in patients with CBL without increasing adverse reactions. [6]

## Figures and Tables

**Table 1:** Comparison of clinical effects between the two groups of patients (*n*, (%)).

Group	Number of cases	Effective	Valid	Invalid	Total efficiency
	55	18 (32.73)	20 (36.36)	17 (30.91)	38 (69.09)
Control group	55	29 (52.73)	18 (32.73)	8 (14.55)	47 (85.46)
*χ* ^2^					4.193
*P*					0.041

**Table 2:** Comparison of arrhythmia between the two groups (*n*, $\bar{x}$ ± *s*, times).

Group	Number of cases	*Paroxysmal atrial fibrillation*		*Atrial precontraction*		*Premature ventricular contraction*	
		Before the treatment	4 weeks after treatment	Before the treatment	4 weeks after treatment	Before the treatment	4 weeks after treatment
Control group	55	273.62 ± 32.22	86.64 ± 20.86^a^	4973.89 ± 491.31	1157.67 ± 204.49^a^	8241.31 ± 808.45	1414.87 ± 350.16^a^
Combined group	55	279.82 ± 31.67	58.85 ± 18.78^a^	5086.05 ± 401.38	767.47 ± 186.00^a^	8219.25 ± 935.02	894.85 ± 360.60^a^
*T*		1.018	7.341	1.311	10.469	0.132	7.673
*P*		0.311	0.001	0.193	0.001	0.895	0.001

**Table 3:** Comparison of plasma viscosity between the two groups (*n*, $\bar{x}$ ± *s*).

Group	Number of cases	*Whole blood low shear viscosity value (mpa·s * ^*−1*^)		*Whole blood high-shear viscosity value (mpa·s * ^*−1*^)		*Fb (ρ/g·L * ^*−1*^)	
		Before the treatment	4 weeks after treatment	Before the treatment	4 weeks after treatment	Before the treatment	4 weeks after treatment
Control group	55	10.43 ± 1.15	8.76 ± 1.30^a^	6.61 ± 1.15	5.13 ± 0.85^a^	370.32 ± 37.10	331.68 ± 23.75^a^
Combined group	55	10.34 ± 1.44	7.22 ± 1.64^a^	7.01 ± 1.64	4.81 ± 0.70^a^	370.48 ± 40.18	292.98 ± 25.01^a^
*t*		0.349	5.474	1.477	2.142	0.021	8.320
*P*		0.727	0.001	0.143	0.034	0.983	0.001

^a^indicates comparison with the same group before treatment, ^a^*P* < 0.05.

**Table 4:** Comparison of the vascular endothelial function between the two groups of patients (*n*, $\bar{x}$ ± *s*).

Group	Number of cases	*NO (μg/L)*		*ET-1 (pg/L)*		*vWF (%)*	
		Before the treatment	4 weeks after treatment	Before the treatment	4 weeks after treatment	Before the treatment	4 weeks after treatment
Control group	55	38.95 ± 6.03	49.52 ± 5.42^a^	75.86 ± 10.08	58.00 ± 7.11^a^	172.41 ± 19.88	130.60 ± 20.14^a^
Combined group	55	38.81 ± 5.17	59.51 ± 6.96^a^	72.90 ± 9.98	49.43 ± 7.49^a^	176.22 ± 28.38	118.90 ± 12.50^a^
*t*		0.128	8.399	1.547	6.153	0.816	3.66
*P*		0.899	0.001	0.125	0.001	0.416	0.001

*Note*.^a^ indicates comparison with the same group before treatment ^a^*P* < 0.05.

**Table 5:** Comparison of the total incidence of adverse reactions between the two groups (*n*, (%)).

Group	Number of cases	Vomiting	Lack of appetite	Nervous system damage	dry mouth	Diarrhea	Nausea	Overall incidence of adverse reactions
Control group	55	2 (3.64)	3 (5.45)	1 (1.82)	1 (1.82)	1 (1.82)	1 (1.82)	9 (16.36)
Combined group	55	1 (1.82)	1 (1.82)	0(0.00)	1 (1.82)	1 (1.82)	1 (1.82)	5 (9.09)
*χ* ^2^								1.310
*P*								0.252

## Data Availability

The raw data supporting the conclusion of this article will be available by the authors without undue reservation.
